The article "An Effective and Lightweight Deep Electrocardiography Arrhythmia Recognition Model Using Novel Special and Native Structural Regularization Techniques on Cardiac Signal" was retracted in 2023. Reasons: unreliable results or conclusions; concerns about the data; concerns about the peer review; concerns about the citations.

# An Effective and Lightweight Deep Electrocardiography Arrhythmia Recognition Model Using Novel Special and Native Structural Regularization Techniques on Cardiac Signal

**DOI:** 10.1155/2022/3408501

**Published:** 2022-04-12

**Authors:** Hadaate Ullah, Md Belal Bin Heyat, Hussain AlSalman, Haider Mohammed Khan, Faijan Akhtar, Abdu Gumaei, Aaman Mehdi, Abdullah Y. Muaad, Md Sajjatul Islam, Arif Ali, Yuxiang Bu, Dilpazir Khan, Taisong Pan, Min Gao, Yuan Lin, Dakun Lai

**Affiliations:** ^1^School of Materials and Energy, State Key Laboratory of Electronic Thin Films and Integrated Devices, University of Electronic Science and Technology of China, Chengdu 610054, Sichuan, China; ^2^IoT Research Center, College of Computer Science and Software Engineering, Shenzhen University, Shenzhen 518060, Guangdong, China; ^3^International Institute of Information Technology, Hyderabad, Telangana 500032, India; ^4^Department of Science and Engineering, Novel Global Community Educational Foundation, Hebersham, NSW 2770, Australia; ^5^Department of Computer Science, College of Computer and Information Sciences, King Saud University, Riyadh 11543, Saudi Arabia; ^6^Department of Orthopedics Surgery, West China Hospital, Sichuan University, Chengdu 610041, Sichuan, China; ^7^School of Computer Science and Engineering, University of Electronic Science and Technology of China, Chengdu, Sichuan, 610054, China; ^8^Computer Science Department, Faculty of Applied Sciences, Taiz University, Taiz 6803, Yemen; ^9^Faculty of Medicine, Perm State Medical University, Perm 614000, Russia; ^10^Department of Studies in Computer Science, University of Mysore, Mysore, Karnataka, India; ^11^IT Department, Sana'a Community College, Sana'a 5695, Yemen; ^12^College of Computer Science, Data Intelligence and Computing Art Lab, Sichuan University, Chengdu 610065, China; ^13^Department of Computer Science, University of Science and Technology, Bannu, Pakistan; ^14^Biomedical Imaging and Electrophysiology Laboratory, School of Electronic Science and Engineering, University of Electronic Science and Technology of China, Chengdu 610054, Sichuan, China

## Abstract

Recently, cardiac arrhythmia recognition from electrocardiography (ECG) with deep learning approaches is becoming popular in clinical diagnosis systems due to its good prognosis findings, where expert data preprocessing and feature engineering are not usually required. But a lightweight and effective deep model is highly demanded to face the challenges of deploying the model in real-life applications and diagnosis accurately. In this work, two effective and lightweight deep learning models named Deep-SR and Deep-NSR are proposed to recognize ECG beats, which are based on two-dimensional convolution neural networks (2D CNNs) while using different structural regularizations. First, 97720 ECG beats extracted from all records of a benchmark MIT-BIH arrhythmia dataset have been transformed into 2D RGB (red, green, and blue) images that act as the inputs to the proposed 2D CNN models. Then, the optimization of the proposed models is performed through the proper initialization of model layers, on-the-fly augmentation, regularization techniques, Adam optimizer, and weighted random sampler. Finally, the performance of the proposed models is evaluated by a stratified 5-fold cross-validation strategy along with callback features. The obtained overall accuracy of recognizing normal beat and three arrhythmias (V-ventricular ectopic, S-supraventricular ectopic, and F-fusion) based on the Association for the Advancement of Medical Instrumentation (AAMI) is 99.93%, and 99.96% for the proposed Deep-SR model and Deep-NSR model, which demonstrate that the effectiveness of the proposed models has surpassed the state-of-the-art models and also expresses the higher model generalization. The received results with model size suggest that the proposed CNN models especially Deep-NSR could be more useful in wearable devices such as medical vests, bracelets for long-term monitoring of cardiac conditions, and in telemedicine to accurate diagnose the arrhythmia from ECG automatically. As a result, medical costs of patients and work pressure on physicians in medicals and clinics would be reduced effectively.

The article "An Effective and Lightweight Deep Electrocardiography Arrhythmia Recognition Model Using Novel Special and Native Structural Regularization Techniques on Cardiac Signal" was retracted in 2023. Reasons: unreliable results or conclusions; concerns about the data; concerns about the peer review; concerns about the citations.

## 1. Introduction

Cardiovascular disease (CVD) is one of the leading human life-threatening disease; with around 17.7 million people lose their lives due to CVDs annually [1]. The mortality and prevalence of CVDs are still on rise in worldwide, therefore continuous monitoring of heart rhythm is becoming a crucial issue to prevent and control the CVDs. Arrhythmia is common rhythm but a complex CVD that leads other heart diseases. ECG is the primary medical diagnostic tool for CVD in practice and provides a comprehensive picture of patient's cardiac conditions. Currently, physicians perform post hoc analysis through ECG waveforms to diagnose whether a patient is well or sick, which is inefficient, time-consuming, and also not so reliable due to the factors of physicians' experience and expertise level. Computer-aided automatic ECG analysis could effectively enhance the diagnosis efficiency as well as shorten diagnosis time. Nowadays, automatic arrhythmia recognition systems are becoming more essential to diagnose the heart diseases. It is more useful in wearable or portable devices. The basis of a traditional automatic system is to extract features correctly and then classify or diagnose with a shallow machine learning approach. A traditional automatic ECG arrhythmia recognition system usually comprises of four parts: (1) preprocessing [2]; (2) beat segmentation [3]; (3) feature extraction such as QRS width finding [4], R-R intervals [5], and wavelet transform [6]; and (4) classification algorithms such as support vector machine (SVM) [7], genetic algorithm (GA) for SVM optimization [8], artificial neural network (ANN) [9], and random forest (RF) [10]. After extracting the features, sometimes feature selection techniques such as linear discriminant analysis (LDA) [6], independent component analysis (ICA) [5, 6], and principal component analysis (PCA) [6, 9, 11] are needed to alleviate the dimensions and dispel the related features to enhance the accuracy. Recently, Jha and Kolekar [12] proposed an efficient ECG arrhythmia classification approach using the tunable Q-wavelet transform and SVM classifier to detect the normal and seven types of arrhythmias, where ECG beats were decomposed up to the level of sixth. The achieved average accuracy, sensitivity, and specificity are 99.27%, 96.22%, and 99.58%, respectively, for eight different beat classes. Abdalla et al. [13] also presented a complete ensemble nonstationary and nonlinear decomposition method to extract the features of ECG beats with intrinsic mode functions (IMFs), where four parameters (coefficient of dispersion, singular values, average power, and sample entropy) were computed from first six IMFs to construct the features' vector. Their received average accuracy, sensitivity, and specificity are 99.9%, 99.7%, and 99.9%, respectively, to identify the normal and four different arrhythmias. An automatic heartbeat classification method was addressed by Mondéjar-Guerra et al. [14] with the combination of multiple SVMs to classify the normal and three abnormal beats and achieve satisfactory results, where various descriptors (LBP-local binary patterns, HOS-higher order statistics, and several amplitude values) based on wavelets were employed to extract the morphological and temporal characteristics of ECG beats. Sometimes, ensemble or hybrid methods in shallow machine learning algorithms are developed to achieve better predictive performance than the constituent learning algorithms alone [15–17]. Although many shallow machine learning methods, for examples [12–14], have been proposed to classify ECG arrhythmia with good findings and encouraging results, they are still facing challenges in feature extraction using engineering techniques as well as dealing the imbalanced data [18, 19]. Several researchers have tried to solve the issue by optimizing the classifiers with the generalization capabilities [20–29]. In the conventional methods, learning parameters during training the proposed techniques are able to cover multiple features with the confined nonlinear fitting and approximated capabilities in the facing of complex ECG waveforms. So, in the training of big data-driven context, the classification efficiency of conventional classifiers is not satisfactory [30].

The article "An Effective and Lightweight Deep Electrocardiography Arrhythmia Recognition Model Using Novel Special and Native Structural Regularization Techniques on Cardiac Signal" was retracted in 2023. Reasons: unreliable results or conclusions; concerns about the data; concerns about the peer review; concerns about the citations.

In contrast, recent deep learning approaches could offer the solutions to overcome the challenges of shallow machine learning algorithms performing feature learning automatically [31–34] followed the human brain structure. These approaches usually combine feature extraction and classification steps of traditional methods, optimize them with the sufficient amount of data, and provide good interpretability. Besides, deep learning concepts play a vital role at present because acquired ECG data in medical and clinics are enlarged day by day, around more than 300 million ECGs are preserved worldwide annually [34, 35]. More data are helpful in the deep learning models for handling the large number of variables during training. Therefore, nowadays, it is becoming a difficult task to analyze the ECG beat-by-beat with the traditional techniques, especially in the wearable health monitoring circumstances. Hence, engineers and researches are shifting their concentrations on beat classification studies with the deep learning approaches. The reported findings in the literature [36–42] show that with the different layer initialization strategies and some promising techniques such as k-fold cross-validation, stratified k-fold cross-validation, regularization techniques (dropout [36] and batch normalization (BN) [37]), and Adam optimizer [38] in deep learning networks perform such good job. Deep neural networks (DNNs) [39, 43], CNN [40], long short-term memory (LSTM) [41], recurrent neural networks (RNNs) [40], and also merging of these approaches [42] were employed to classify the ECG arrhythmia. Hannun et al. [39] developed an end-to-end approach in deep learning to identify the 12 classes of ECG rhythms from 53,549 patients with 91,232 single-leads monitoring device in ambulatory condition. Their achieved results validated with a consensus board committee of certified practicing cardiologists and findings demonstrated that the deep learning approach is able to classify 12 distinct rhythms with a good performance approximately same to that of cardiologists. It states that deep learning approaches could reduce the misdiagnosed rate of computerized interpretations and enhance the efficiency of cardiologists in urgent circumstances. RNNs and LSTM are mainly emerged for sequential analysis of data and a great progress of deep learning due to its successful adaptations of various versions in the basic architecture depending on the applications. Yildirim [41] presented a deep bidirectional LSTM (DBLSTM) based on the wavelet sequences of input data to classify five different heartbeats from the MIT-BIH arrhythmia dataset and experimental results provide the recognition accuracy of 99.39%. CNNs are the hierarchical neural networks where convolutional layers are changed with the subsampling of layers and reminiscent of complex and simple cells similar to the human visual cortex [44] following the fully connected layers, which are same as multilayer perceptron (MLP). CNNs are commonly employed in deep learning for object detection from complex images, achieving high accuracy results compared with the state-of-the-arts methods [45]. Recently, it is widely used in anomaly detection and ECG classification. Among the various categories of deep learning models, CNN is a more promising technique due to its good detecting capability of vital features from the raw information at the various levels of networks automatically without any human supervision. The raw ECG signals usually belong to 1D data features. CNN allows its input as the multidimensional (1D, 2D, and 3D) forms that narrate the attributes of raw signal. Kiranyaz et al. [46] proposed a patient-specific arrhythmia classification approach with 1D convolutional neural network in real time, which could be utilized to identify long ECG streams of patients with a wearable device. Some attractive works with 1D CNNs [46–48] are introduced to identify the arrhythmia from the ECG signals but the received performance results are not so satisfactory. The factors behind such performance are as follows: (i) 1D CNN is less versatile, and (ii) it does not attain the intended aim of attainment [49]. In contrast, 2D CNN is a promising approach that could handle such types of oversights in 1D CNN due to the representing of time-series data in 2D format as the input. And hence, we have chosen 2D CNN for our study, where 2D transformations of raw time-series data are performed to make it suitable as the input of 2D CNN. The more vital information can be achieved in 2D CNN compared to 1D CNN that helps to improve the accuracy easily [50], herein the authors first extract PQRST features of a single heartbeat from the raw ECG signals after some preprocessing. In [51, 52], it was reported that image-based 2D CNN arrhythmia classification structures obtain better performance compared to 1D CNN, where time domain ECG signals belonging to the heartbeats were transformed into 2D time frequency spectrograms by STFT (short time Fourier transform) to be compatible with the input of their proposed 2D CNN model. The raw ECG signals from the MIT-BIH arrhythmia dataset were first segmented into the heartbeats and then transformed into 2D gray-scale images, which were used as the input of 2D CNN architecture [53, 54] and achieved satisfactory results for identifying the heartbeats. Recently, Ullah et al. [55] proposed a 2D CNN model to classify the heartbeats from the raw ECG signals of MIT-BIH arrhythmia dataset and the performance is compared to the 1D CNN, where the experimental results demonstrate that the performance of their proposed 2D CNN model is better than 1D CNN. Therefore, 2D CNN is more feasible to diagnose arrhythmia from the ECG signals.

The article "An Effective and Lightweight Deep Electrocardiography Arrhythmia Recognition Model Using Novel Special and Native Structural Regularization Techniques on Cardiac Signal" was retracted in 2023. Reasons: unreliable results or conclusions; concerns about the data; concerns about the peer review; concerns about the citations.

Moreover, although several 2D CNN approaches [49–55] have achieved impressive results to detect the arrhythmia from the ECG signal with good accuracy, a 2D CNN model with superior accuracy, guaranteed data imbalance problem-solving, and a lightweight end-to-end 2D deep learning model is more essential for real-life applications. Meanwhile, an imbalanced dataset would decline the overall accuracy of the model and result in diagnosis errors of the diseases, because a small increase in accuracy has a great impact on the diagnosis [56, 57]. In this study, two deep learning models, namely Deep-SR and Deep-NSR, based on 2D CNN approaches were proposed, which are more effective(superior accuracy), efficient (lightweight), and generalized that alleviate the data imbalance problem than the state-of-the-art models to recognize the arrhythmias in practical life. The major factors behind such satisfactory results are as follows: (i) proper model designing with proper initialization of layers and usage of some diverse regularization techniques such as BN [37] and dropout [36], and (ii) usage of weighted random sampler [58], Adam optimizer [38], and early stopping [59] in the developed model training module. The Deep-NSR is lightweight compared to Deep-SR; it is more applicable than Deep-SR for deploying in real-life applications. In the proposed Deep-NSR, (i) the adaptive pooling layer is directly connected to the softmax layer and has no dropout and fully connected layers, and (ii) the number of kernels or filters in the last convolution layer is equal to the number of target classes following the structural regularization technique [60]. As a result, the total learnable parameters are drastically reduced in the designed model and play an impact to the size of model. So far we are concerned; it is the first attempt to apply the structural regularization concept [60] in a model to diagnose ECG arrhythmia diseases that drastically reduce the learnable parameters in a model which results in a lightweight model as well as a low computational cost.

The article "An Effective and Lightweight Deep Electrocardiography Arrhythmia Recognition Model Using Novel Special and Native Structural Regularization Techniques on Cardiac Signal" was retracted in 2023. Reasons: unreliable results or conclusions; concerns about the data; concerns about the peer review; concerns about the citations.

To the end, the major contributions are as follows:

- Two lightweight 2D CNN models are developed compared to the state-of-the-art 2D CNN models to identify the ECG arrhythmia, which could be more useful in real-life applications to diagnose the diseases automatically.
- Any handcrafted feature extraction technique is not required in this study.
- A state-of-the-art improvement in performance is acquired for both proposed models with the 2D transformed images as the input of deep models in ECG arrhythmia classification, which expresses high model generalization.
- The achievement of model performance is due to the usage of several diverse regularization techniques (BN [37] and dropout [36]), Adam optimizer [38], weighted random sampler [58], early stopping [59], on-the-fly data augmentation [61], and proper initialization of layers [62, 63] in the designed models. As such, data imbalance shortcoming on the publicly available datasets, even on clinical or own producing data, could be overcome.

The rest of the article is organized as follows: The proposed methods and materials are demonstrated in Section 2 with details. Results with discussion are illustrated in Section 3. Finally, a conclusion with some future directions is provided in Section 4.

## 2. Materials and Methods

The whole architecture of our proposed system in ECG arrhythmia classification is depicted in Figure 1. In this study, we have used a benchmark dataset MIT-BIH arrhythmia database [64] to train and test the proposed models. First, ECG signals from this dataset are transformed into two-dimensional 128 × 128 RGB images in the preprocessing step that are fed as the input of our proposed models. Among the fourteen annotated beat and three non-beat types in the MIT-BIH arrhythmia database, we have considered the class mappings based on AAMI recommendation, which is expressed as (i) N-normal (N-normal, R-right bundle branch block, L-left bundle branch block, e-atrial escape, and j-nodal (junctional) escape), (ii) V-ventricular ectopic (E-ventricular escape and V-premature ventricular contraction), (iii) S-supraventricular ectopic (a-aberrated atrial premature, S-supraventricular premature, J-nodal (junctional) premature, and A-Atrial premature), (iv) F-fusion (fusion of normal and ventricular), and (v) Q-unknown (/-Paced, Q-unclassified, and f-fusion of normal and paced). Herein, Q class is not taken into account due to the involvement of paced and unclassified beats. So, our proposed models have performed recognition on the total four types of beats identified as N, S, V, and F classes in the classification step. The overall system consists of the following three subsections: (i) data preprocessing, (ii) feature extraction and classification based on the proposed CNN models, and (iii) model evaluation.

The article "An Effective and Lightweight Deep Electrocardiography Arrhythmia Recognition Model Using Novel Special and Native Structural Regularization Techniques on Cardiac Signal" was retracted in 2023. Reasons: unreliable results or conclusions; concerns about the data; concerns about the peer review; concerns about the citations.

### 2.1. Dataset Description and Acquisition

The MIT-BIH arrhythmia benchmark dataset [64] contains a total of 48 records from 47 patients, where 25 are men of age 32–89 and 22 women of age 23–89, two-channel ECG recordings, the sampling rate is 360 Hz and each record has a duration of half an hour. The resolution of digitization for each recording is 11-bit over a 10 mV range. The dataset is established by the MIT lab and Beth-Israel Hospital in Boston. In most records of the dataset, the upper signal is MLII (a modified limb lead II) while the lower signal is modified lead V1 (seldom V2 or V5 and V4 in one instance), all are placed on the chest [64]. QRS complexes of normal ECG signal are commonly noticeable in the upper signal lead II based on the website located at https://www.physionet.org for the dataset. So, we have chosen the lead II signal in our experiment. Records 102 and 104 are involved with the surgical dressings of patients, and records 102, 104, 107, and 217 have the involvements of paced beats, so we have eliminated these records in our experiment.

### 2.2. Data Preprocessing

Here, each ECG record is transformed into its equivalent RGB images after segmentation of each ECG beat from all the records of dataset. In the dataset, each record has three files which are annotation, signals, and header files. First, the dataset is downloaded manually from https://physionet.org/content/mitdb/1.0.0/. Then annotation file is accessed and processed with the Glob module of python and WFDB Toolbox. After reading the annotation of all records from the dataset, the data for each beat are sliced with the sampling frequency of 360 Hz. Herein, segmentation is accomplished by detecting the R peaks from all records with the help of Python Biosppy module and forming a CSV file with a sequence of the heartbeats for each beat type. Pan and Tompkins algorithm [65] for R-peak detection is well commenced and comparatively more accurate as well as arrhythmia is mainly labeled at the peak of each R-peak wave. And hence, this R peaks detection technique is chosen in this study. Once the R-peaks are detected to segment a beat, the present and next R peaks are also considered and have taken half of the distance of those, the included signals represent a segmented beat. A similar process is maintained for the segmentation of all beats. For transforming the segmented beats into the beat images, OpenCV and Matplotlib modules of python are employed. Finally, we have got a total of 97720 images of 128 × 128 scale size from the MIT-BIH arrhythmia dataset for four-beat types. The obtained beat images are fed into our automatic deep-based feature extractor models as the input to extract the local area-specific features by mapping the subtle spatial change of beat images. Then a high-level feature vector is formed from the extracted features. Next, the recognition of beats is performed with the softmax classifier based on this vector, which ensures the summation of the class label scores is 1.

The article "An Effective and Lightweight Deep Electrocardiography Arrhythmia Recognition Model Using Novel Special and Native Structural Regularization Techniques on Cardiac Signal" was retracted in 2023. Reasons: unreliable results or conclusions; concerns about the data; concerns about the peer review; concerns about the citations.

The augmentation of input images of the models for the training set could provide the benefit of less over-fitting dealing with class imbalance problems. Our proposed models receive 2D beat images as the input, so we can easily resize, rotate, and crop the images in the training module that do not degrade the model's performance but increase the training data numbers and may help to alleviate the over-fitting of models maintaining equal distribution among the classes. To maintain the equal distribution of classes, it is particularly so essential in medicals and clinics to diagnosis the diseases accurately through data analysis. Most data in medicals and clinics are normal and only a few numbers of data are abnormal. Some anterior arrhythmia works performed augmentation manually but herein we have performed online augmentation on-the-fly [61] of images. The major benefits of this concept are hassle-free and time-saving unlike manual augmentation. In this work, beat images are rotated randomly at a maximum of 6 degrees. Then the augmented images are resized into a 64 × 64 scale size before converting it into tensors inside the model to speed up the learning. The augmentation in a model usually provides better results compared to nonaugmented data [52, 53].

### 2.3. Feature Extraction Based on the Proposed CNN Models and CNN Classifier

In this study, we have developed two 2D CNN models, where convolutional and pooling layers are more compatible to the spatial locality of a filter for extracting the features from an image. A competition on ImageNet Large Visual Perception Challenge (ILSVRC) [66] has found some successful developed CNN models such as AlexNet [45], GoogleNet [67], and VGGNet [68], which are widely shown in the computer vision field. ResNet [69], and DenseNet [70] are also interesting CNN models as the deeper networks, recently appeared in image classification. In our developed CNN models, we have used some basic structures of AlexNet and VGGNet. So, the performance of our proposed models is compared to AlexNet and VGGNet. Our transformed beat images are relatively simple backgrounds of 128 × 128 sized RGB images. Therefore, high depth layers are not needed to optimize the proposed models, which may cause over-fitting and subsequently might degrade the model performance. Figures 2 and 3 demonstrate end-to-end internal layer architecture of the proposed Deep-SR model and Deep-NSR model, respectively. Careful consideration has been taken to determine the depth and organization of relevant layers. This is very crucial to recognize the transformed beat images correctly without any over-fitting of the proposed models from a small dataset due to the lack of a sufficient number of samples.

The article "An Effective and Lightweight Deep Electrocardiography Arrhythmia Recognition Model Using Novel Special and Native Structural Regularization Techniques on Cardiac Signal" was retracted in 2023. Reasons: unreliable results or conclusions; concerns about the data; concerns about the peer review; concerns about the citations.

The first proposed model is comprised of five convolution blocks, one maxpooling layer, and one average pooling layer to capture the area-specific features and followed by a fully connected layer or linear layer to classify the arrhythmia. After each convolution layer, a nonlinear activation function rectified linear unit (ReLU) is used to alleviate the vanishing gradient problem usually generated from the output range of activation function during gradient computation loss in the back-propagation step. It helps the optimizer to receive the optimal set of weights quickly and results are a faster convergence of stochastic gradient descent and low computational cost. Let *x*^*i*^ and *y*^*j*^ represent the *i*^th^ input and *j*^th^ output feature map of a convolutional layer, respectively, then activation function employed in CNNs could be expressed as under:

(1) $$\begin{array}{c} y^{j}=\max\left(0,b^{j}+\underset{i}{\sum }z^{ij}*x^{i}\right), \end{array}$$

where *z*^*ij*^ indicates the convolutional filters between *x*^*i*^ and *y*^*j*^, and *b*^*j*^ represents the bias. The symbol *∗* expresses the convolutional operation.

If a layer has *M* input and *N* output maps, then it will hold *N* 3D filters of size *d* × *d* × *M*, where *d* × *d* signify the size of local receptive fields as well as every filter has its own bias. In the later, it is addressed as max (*x*, 0) since ReLU allows only values above of zero analogous to its biological counterpart of action potential. This feature of ReLU allows resolving the nonlinear problems of the models. After each ReLU, batch normalization (BN) layer has been employed to accelerate the training. As a result, the learnable parameters are converged at the earliest possible training time providing better accuracy [37]. It also reduces the internal covariate shift and the sensitivity of training toward weight initialization. This is one kind of regularization technique to cut down the over-fitting in the training phase. The relevant features from our preprocessed images are mainly extracted by the convolutional layers in the proposed models. The convolutional layers are the prime components of CNNs, where major functions of CNNs are performed. The operation of a convolutional layer is expressed as under:

(2) $$\begin{array}{c} y=f\left(\sum_{i=1}^{n}\theta_{i}^{T}x_{i}+b\right). \end{array}$$

Here *θ* and *b* indicate the weight and bias parameters of the layer, and *f* (.) represents the activation function.

The article "An Effective and Lightweight Deep Electrocardiography Arrhythmia Recognition Model Using Novel Special and Native Structural Regularization Techniques on Cardiac Signal" was retracted in 2023. Reasons: unreliable results or conclusions; concerns about the data; concerns about the peer review; concerns about the citations.

We have tested the first convolution layer with 5 × 5 kernel size, 32 kernels, 2 strides, false bias, and other parameters such as dilation and padding as default. The remaining four convolution layers are with 3 × 3 kernel size, false bias, and other parameters as default, and subsequently 64, 128, 256, and 512 kernels for the second, third, fourth, and fifth convolution layers, respectively. Large filter size at the starting with spatial down-sampling by convolution of striding 2 and a successive maxpooling with stride of 2 are employed to suppress the irrelevant features from the images. In the ECG beat images, the relevant features remain in the small part of the whole image. The subsequent convolution layers with small size and no spatial down-sampling can easily extract locally repeating features and reduce the computational cost. Pooling layers (maxpooling and average pooling) are operated independently on every depth slice of the input and act as the translation-invariant, which compute a fixed function of the input volume with some hyperparameters and have no learnable parameters. So, pooling layers are also called subsampling layers and alleviate the resolution of feature maps on the inputs. Here, after the first convolution layer, only a maxpooling layer with the kernel size of 3 × 3 and the stride of 2 is added to reduce the spatial dimension of the feature map. It helps to control the over-fitting of the models by decreasing the learnable parameters in the subsequent convolution layers. Extractions of global features related to the pixel of neighborhood are accomplished with the maxpooling and convolution. The maxpooling operation in this study enumerates the maximum value as a set of neighboring inputs. The pooling of feature map in a layer can be expressed as follows:

(3) $$\begin{array}{c} P_{i}^{1,j}=\underset{r\in R}{\max}\left(c_{i\times T+r}^{1,j}\right), \end{array}$$

where *T* indicates pooling stride and *r* represents pooling window size. The average pooling layer with the size of 3 × 3 and the stride of 2 is added just before the last convolution block to extract the average spatial high-level features and it provides an output shape of 11 × 11. After bypassing four convolution blocks, maxpooling, and average pooling layers, the output shape of the last convolution block is reduced to 9 × 9. Finally, the adaptive average pooling reduces the dimension of the tensors so that they might be fitted into the fully connected layer.

The article "An Effective and Lightweight Deep Electrocardiography Arrhythmia Recognition Model Using Novel Special and Native Structural Regularization Techniques on Cardiac Signal" was retracted in 2023. Reasons: unreliable results or conclusions; concerns about the data; concerns about the peer review; concerns about the citations.

The dropout layer [36] is also a regularization method, which reduces over-fitting by alleviating the dependency between the layers introduced by Hinton. It excludes some neurons from learning in the training phase that helps to prevent over-fitting. It randomly sets its input units 0 to 1. In this study, we have used a dropout layer with the probability of 0.3 and its location just before the fully connected layer. Usually, it is not used in the convolutional blocks to maintain the co-adaptation between the nodes. The high-level decision of the model has appeared at the output end of fully connected layer, which can be considered as the classification phase. Each neuron herein is linked to all activations of the previous layers. This layer reads up the feature vector for the softmax layer to classify accurately, whereas the earlier layers carry out the feature learning. Finally, a softmax layer is added at the end of the models to classify the arrhythmia labels with a numerical processing. It is extensively employed in machine learning as well as deep learning. The function can be defined as below:

(4) $$\begin{array}{c} y^{\left(i\right)}=\frac{\exp\left(z^{\left(i\right)}\right)}{\sum_{j-1}^{C}\exp\left(z^{\left(j\right)}\right)}, \end{array}$$

where *z*^(*i*)^ is the last output vector of fully connected layer and fed to the softmax layer to measure the probability, *y*^(*i*)^ of each beat class, *C* is the total number of beat classes, and *i* indicate the class index.

The complete weights are learned with the gradient-based back-propagation algorithm. A series of convolution layers with batch BN and ReLU layers and pooling layers provides the screening of high-level features from the desired areas of beat images. The architecture with the hyperparameters of the Deep-SR model is illustrated in Table 1. The above explanation for all layers of Deep-SR model is also applicable for Deep-NSR model. The difference is in the last convolution layer. First, the number of the kernel is equal to the number of class label numbers instead of 512. Second, the adaptive average pooling layer is directly connected to the softmax layer through the fully connected layer and has no dropout layer. This technique is called the native structural regularized method in CNN [60] and applied as the first on 2D CNN to detect ECG arrhythmia. As a result, the total number of model learnable parameters is drastically reduced and the model size become too small in comparison with the Deep-SR model. This technique helps to alleviate model over-fitting and accelerate the training as well as enhance the model efficiency. The architecture with the hyperparameters of the Deep-NSR model is given in Table 2.

The article "An Effective and Lightweight Deep Electrocardiography Arrhythmia Recognition Model Using Novel Special and Native Structural Regularization Techniques on Cardiac Signal" was retracted in 2023. Reasons: unreliable results or conclusions; concerns about the data; concerns about the peer review; concerns about the citations.

### 2.4. Cost Function and Evaluation Metrics

The cross-entropy loss or cost functions in equations (5)–(7) measure how well the model is trained and receives the differentiation between the training sample and predicted output to calculate the training loss. The loss function might be alleviated through the optimizer function, which is more adaptable for high-class imbalanced data compared to other available loss functions.

(5) $$\begin{array}{c} \text{loss}\left(x,\text{class}\right)=-\log\left(\frac{\left(\exp\left(x\left[\text{class}\right]\right)\right)}{\sum_{j}\exp\left(x\left[j\right]\right)}\right), \end{array}$$

(6) $$\begin{array}{c} \text{loss}\left(x\text{,class}\right)=-x\left[\text{class}\right]+\log\left(\underset{j}{\sum }\exp\left(x\left[j\right]\right)\right). \end{array}$$

For class weights:

(7) $$\begin{array}{c} \text{loss}\left(x\text{,class}\right)=\text{wieght}\left[\text{class}\right]\left(-x\left[\text{class}\right]+\log\left(\underset{j}{\sum }\exp\left(x\left[j\right]\right)\right)\right). \end{array}$$

The above cost function is the combination of equations (8)–(10). Here *x* is the output of the fully connected layer and it is fed to the input function of softmax classifier that acts as the normalized score for each class. If the number of classes is *C*, then each class represents the index in the range [0, *C* − 1]. The model is trained on a mini-batch of the training samples and *x* is in range (mini-batch, *C*). In the case of a mini-batch, the losses are averaged across all samples within it. The log softmax function is computed based on the following equation:

(8) $$\begin{array}{c} \log\;\mathrm{soft}\;\max\left(x_{i}\right)=\log\left(\frac{\exp\left(x_{i}\right)}{\sum_{j}\exp\left(x_{j}\right)}\right). \end{array}$$

Here *x*_*i*_ is the *i*^th^ dimension of output tensors in which the Log SoftMax function is computed. The negative log-likelihood loss is defined by the following equation:

(9) $$\begin{array}{c} \text{nllloss}\left(x\text{,}y\right)=L\\ =\left\{l_{1},l_{2},\ldots ,l_{n}\right\},\\ \text{ln}=-\left(w_{y_{n}}x_{n,y_{n}}\right). \end{array}$$

For unreduced loss:

(10) $$\begin{array}{c} \text{nllloss}\left(x\text{,}y\right)=\left\{\begin{array}{c} \sum_{n=1}^{N}\frac{1}{\sum_{n=1}^{N}w_{y_{n}}}\ln\;\text{if reduction}={}^{\prime }\text{mean}{}^{\prime },\\ \sum_{n=1}^{N}\ln\;\text{if reduction}={}^{\prime }\text{sum}{}^{\prime }. \end{array}\right. \end{array}$$

Here *N* is the batch size.

The article "An Effective and Lightweight Deep Electrocardiography Arrhythmia Recognition Model Using Novel Special and Native Structural Regularization Techniques on Cardiac Signal" was retracted in 2023. Reasons: unreliable results or conclusions; concerns about the data; concerns about the peer review; concerns about the citations.

In this study, we have considered three performance metrics for the evaluation of our proposed models on the MIT-BIH dataset that is highly imbalanced. The exactness and sensitivity of a model are measured by precision and recall, respectively. The unweighted average F_1-score_ (UAF_1_) captures the accuracy on class imbalance by summing up the UAF_1_ calculated on precision and recall for each predicted class sample, then divided by the number of classes to reduce the biasing of large classes samples. The unweighted average recall (UAR) measures the sensitivity of the models based on the recall of each predicted class sample that represents the balanced accuracy to reduce the impact of unbalanced class bias. These two metrics are suitable for the classification of unbalanced classes. The standard accuracy is measured based on the total true positive (TP) and true negative (TN) samples out of the total number of samples. The matrices are measured by the following equations [23, 71–73]:

(11) $$\begin{array}{c} \text{Precision}=\frac{\text{TP}}{\text{TP}+\text{FP}},\\ \text{Recall}=\frac{\text{TP}}{\text{TP}+\text{FN}},\\ {\text{UAF}}_{1}=2\times \frac{\text{precision}\times \text{recall}}{\text{precision}+\text{recall}}\\ =\frac{2\text{TP}}{2\text{TP}+\text{FP}+\text{FN}},\\ \text{UAR}=\frac{\sum \text{per}\_\text{class}\_\text{accuracy}}{c},\\ \text{Accuracy}=\frac{\text{TP}+\text{TN}}{\text{TP}+\text{FP}+\text{TN}+\text{TF}}, \end{array}$$

where TP represents true positive, FP represents false positive, TN represents true negative, FN represents false negative, and *c* is the number of classes.

### 2.5. Implemetation Details

Proposed CNN models are implemented in Python language (version 3.6) with an open-source software library PyTorch [74] framework for deep learning launched by Facebook. Herein, Anaconda 3-5.3.1 provides the Jupyter Notebook facility. Google Tensorboard is applied to visualize the required graphs of various evaluation matrices with the respective CSV files. A GPU-supported computer is essential to reduce the learning time of models. We have employed Core i5-7400 CPU @ 3.00 GHz, 8 GB RAM processor with NVIDIA GeForce RTX 2070 graphic card with 8 GB memory to perform our experiments. With these NVIDIA GPUs, PyTorch is accelerated by CUDA and CUDNN [75]. Some open-source library packages such as Scikit-Learn, Numpy, Pandas, Matplotlib, Wfdb, and Biosspy are also employed to perform the whole work. Herein, at first, the convolution, batch normalization [37], and fully connected layers of proposed models are needed to initialize. The major problem of gradient descent learning algorithm is that it is needed to diverge a model into a local minimum point. So, an intellectual weight initializer is required to achieve the convergence. In CNN, these weights are described as kernels and a group of kernels that form a single layer. In our proposed models, kaiming normal distribution [62] initializes the weights of all the convolution layers. The weight and bias of all batch normalization layers have been initialized with 1 and 0, respectively. Xavier initializer [63] initializes the weights of fully connected layer and bias is initialized with a constant 0. The main worth of these initializers is the balance of gradient scale roughly equivalent in all kernels. We have also excluded the padding procedure to sustain the actual size of images through the convolution and pooling layers. The models' performance with the test data is greatly deflected by altering the ratio of training set and test set. In this study, the whole dataset is divided into a validation set by the random split feature with a given ratio. A validation set is needed to determine either the model is reached at adequate accuracy with the given training set or not. The model is usually falling in over-fitting without a validation set. The random selection mechanism is facing various evaluation effects on a relatively small dataset. K-fold cross-validation is a good evaluation technique to solve such a type of problem. In k-fold, the samples are grouped into the total *k*-fold randomly. If *k* = 10, the samples are grouped into 10-fold randomly and 10 splits have been generated. In each split one fold acts as the testing set and the remaining nine folds act as the training sets. In our work, we have implemented stratified five-fold cross-validation technique. First, we have chosen five-fold to cut down the computational cost and enhance the change of keeping all samples to each fold from each class. Second, we have chosen stratified to ensure the samples from each class to each fold, which alleviates the class imbalance problem of a dataset. Our used MIT-BIH arrhythmia dataset is a class imbalance dataset. The batch size and initial learning rate are set to 64 and 0.0001, respectively. The proposed models are also tested with some other initial learning rates such as 0.001 and 0.00001. But the achieved performance parameters with the initial learning rate 0.001 are better compared to others. This result is due to smooth convergence of the models with this learning rate. The efficient convergence is usually appeared by the internal covariate shift and normalization accelerates and stabilizes the learning process [76]. To optimize the cost function, a gradient descent-based optimizer is utilized with the indicated learning rate. Herein, we have used a stochastic Adam optimizer [38] to receive the better performance compared to some other optimizers such as Adagrad, Adadelta, and stochastic gradient decent (SGD). The learning rate is decreased with the factor of 0.1 if the validation loss is a plateau for five consecutive epochs with the help of learning rate scheduler (REDUCELRONPLATEAU). To ensure the equal representativeness of samples in each class, a weighted random sampler [58] is also chosen in this study. The early stopping [59] regularization is employed to stop the training if the validation loss does not improve for eight consecutive epochs, which helps to receive the optimal training time and reduce the over-fitting. Finally, the acquired overall recognition accuracies are 99.3% and 99.6% for the Deep-SR model and Deep-NSR model, respectively, on four-beat categories.

The article "An Effective and Lightweight Deep Electrocardiography Arrhythmia Recognition Model Using Novel Special and Native Structural Regularization Techniques on Cardiac Signal" was retracted in 2023. Reasons: unreliable results or conclusions; concerns about the data; concerns about the peer review; concerns about the citations.

## 3. Results and Discussion

### 3.1. Performance Analysis of the Proposed Deep-SR and Deep-NSR Models

We have considered the beat samples of four categorical classes (N, S, V, and F) from a benchmark dataset, MIT-BIH arrhythmia based on AAMI. Q class is not considered in this study due to the involvement of unclassified and paced beats. The beat categorization based on AAMI is discussed in detail in Section 2. There are 14 annotated beats and three non-beats in the MIT-BIH arrhythmia dataset. Herein, we have depicted eight transformed beat images in Figure 4 among 14 annotated beats.

An ECG signal usually contains five important waves named as P, Q, R, S, and T. Sometimes, U as the sixth wave may be appeared following T. QRS complex come from Q, R, and S waves. The detection of these waves is a crucial issue in ECG signal analysis for extracting the hidden patterns. In this study, the marked peak value of R wave in the MIT-BIH arrhythmia dataset is utilized as reference point to segment the heartbeats. The R peaks detection is performed by Pan and Tompkins algorithm [65]. After the detection of R peaks, a single beat is considered by taking the half distance of present and next R peaks of detected peak. The characteristics of a normal beat including clinical information is represented in [77]. The drift from the characteristics of a regular beat indicates arrhythmias. The number of beats in each class label is highly imbalanced. To tackle the over-fitting problem due to the high-class imbalance, we have followed and employed the aforementioned strategies and techniques in Section 2.5. The confusion matrix of the proposed Deep-SR model is given in Figure 5, which represents the higher accuracy in each class despite the class imbalance problem in the MIT-BIH arrhythmia dataset indicating the generalization of Deep-SR model. From the confusion matrix, it is observed that the proposed Deep-SR model classifies properly 622 F beats out of 623, 87260 N beats out of 87311, 2697 S beats out of 2706, and 7076 V beats out of 7080. Only 1 F beats, 51 N beats, 9 S beats, and 4 V beats are not classified correctly. The model is converged with a high accuracy due to few catalytic facts such as online augmentation, weighted random sampling, early stopping regularization technique, adaptive learning rate optimization which adjust the weights and cross-entropy loss. From the confusion matrix, it is also evident that the model is unbiased for the different classes. Due to the use of an early stopping regularization scheme, the training of the model is halted if validation loss is not changed in eight consecutive epochs, and the model is evaluated on the test set. The evaluation is performed with the stratified five-fold cross-validation strategy, where the samples are grouped into five folds using stratified sampling, which tries to pick up the samples from each class for reducing the class imbalance problem. Since each fold act as a test set, it is fair strategy to compute the desired metrics.

The article "An Effective and Lightweight Deep Electrocardiography Arrhythmia Recognition Model Using Novel Special and Native Structural Regularization Techniques on Cardiac Signal" was retracted in 2023. Reasons: unreliable results or conclusions; concerns about the data; concerns about the peer review; concerns about the citations.

The model is evaluated on three metrics, namely standard testing accuracy, UAR, and UAF_1_. The results of the respective metrics are depicted in Figure 6(a). The training and testing loss curves are shown in Figure 6(b). From these curves, it is depicted that the training loss curve is declined smoothly and almost stable after nearly 26 epochs, whereas the testing loss curve is abruptly changed initially and becomes stable after around 26 epochs like the training loss curve. This is due to taking time of testing samples to adjust with the trained model at the starting. It is also clear from both curves that the model is halted at 88 epochs due to using early stopping regularization technique. The minimum validation loss, overall accuracy, UAR, and UAF_1_ are 0.0117, 0.9993, 0.9985, and 0.9971, respectively, for the proposed Deep-SR model. A summary of all evaluated metrics from the confusion matrix depicted in Figure 5 is shown in Table 3. The average accuracy, precision, recall, and F_1score_ are 99.96, 99.56, 99.85, and 99.67, respectively. From Table 3, it is obvious that the average values of these metrics are almost same to the overall values represented in Table 4; it represents the generalization of our developed training and testing module for the experiment.

The confusion matrix of the proposed Deep-NSR model is depicted in Figure 7, which represents higher learning unbiased accuracy for ECG arrhythmia classification indicating the generalization of Deep-NSR. From the confusion matrix, it is observed that the proposed Deep-NSR model classifies properly all F beats, 87270 N beats out of 87311, all S beats, and 7078 V beats out of 7080. Only 41 N beats and 2 V beats are misclassified. The results of the desired metrics are depicted in Figure 8(a). The training and testing loss curve are shown in Figure 8(b). From these curves, it is depicted the training loss curve is declined smoothly and almost become stable after nearly 59 epochs while the testing loss curve is abruptly changed initially and become stable after around 59 epochs like the training loss curve. This is due to taking time of testing samples to adjust with the trained model at the starting. It is also clear from both curves that the model is halted at 97 epochs due to early stopping regularization technique. The minimum validation loss, overall accuracy, UAR, and UAF_1_ are 0.0200, 0.9996, 0.9998, and 0.9987, respectively, for Deep-NSR. A summary of all evaluated metrics from the confusion matrix shown in Figure 7 is presented in Table 5. The average accuracy, precision, recall, and F_1score_ are 99.98, 99.76, 99.97, and 99.87, respectively. From Table 5, it is obvious that the average values of all matrices are better than those for Deep-SR, which indicates Deep-NSR will be better to diagnosis the arrhythmias compared to Deep-SR.

The article "An Effective and Lightweight Deep Electrocardiography Arrhythmia Recognition Model Using Novel Special and Native Structural Regularization Techniques on Cardiac Signal" was retracted in 2023. Reasons: unreliable results or conclusions; concerns about the data; concerns about the peer review; concerns about the citations.

From the above analysis, it is evident the behavior and characteristics of both proposed models are similar. The total learnable parameters with size of Deep-SR model and Deep-NSR model are 1573156(16.92 MB) and 399656(11.49 MB), respectively, illustrated in Table 4. The learnable parameters are drastically reduced for the Deep-NSR model compared to Deep-SR, which indicates better model efficiency. As a result, the native structural regularization technique in a model indicates a prosperous concept in ECG arrhythmia detection for real-life applications. Table 4 represents the comparison of evaluation matrices for both models.

### 3.2. Comparison with the State-of-the-Art Models

In this study, we have adopted CNN-based models as the feature extraction and classifier. In 1989, CNN was first commenced by LeCun et al. [78] and flourished by a project for recognizing handwritten zip codes, which resolve the oversights of feed-forward neural networks. With the CNN models, it is possible to extract the interrelation of spatially neighboring pixels and different local features of images through the nonlinear multiple filters. We have compared the performance of our proposed CNN models with the anterior ECG arrhythmia classification tasks. Actually, it is not fully reasonable to directly compare our task with the previous works due to the usage of different strategies as well as different arrhythmia categories. However, Table 6 illustrates the performance comparison of our proposed models to the anterior tasks. From this table, it is evident that our proposed models provide the best results in standard testing accuracy, and UAR compared to previous tasks, which indicates the better effectiveness of our proposed models in ECG arrhythmia recognition. The obtained standard testing accuracy of the proposed Deep-SR and Deep-NSR are 99.93% and 99.96%, respectively. The UAF_1_ is a good evaluation matric for representing the effectiveness of a method on the class imbalance dataset by summing up the precision and recall expressing the exactness and sensitivity of a model at a time. The received UAF_1_ for the Deep-SR model and Deep-NSR model are 99.71% and 99.87%, respectively, as shown in Table 6. The received UAF_1_ on both proposed models represents high generalization and stability compared to the state-of-the-art methods. The UARs are achieved as 99.85% and 99.98% for the Deep-SR and Deep-NSR models, respectively, and surpasses the recall of the state-of-the-art methods, as shown in Table 6. From the comparison (Table 6), it is observed that the traditional machine learning methods with feature engineering techniques provide excellent results in some cases, but (i) it easily tends to over-fitting [34] especially for dealing big data, (ii) it is hard to describe some complex characteristics and high chaos of ECG optimally [79], (iii) high skilled person in this field is required for interpretation the diseases [56], and (iv) more challenges have to be faced for dealing the data imbalance problems [57]. The raw cardiac information from the publicly available datasets or medical/clinics or own developed sensors are usually data imbalance, which has inevitable effect in classification rate. This is due to the lack of availability of some classes and the scoring result is biased toward the dominance classes, which enhances the misclassification rate in machine learning algorithms. In contrast, over-fitting and data imbalance problems in traditional methods could be easily handled for dealing the big data with the deep learning approaches following the techniques and strategies discussed in Section 2.5. As a result, good findings could be achieved with minimum skilled persons in medical and clinics, where ECG data are enlarged day by day, around more than 300 million ECGs are preserved worldwide annually [34, 35]. Large amount of data helps the deep learning approaches to optimize during training. From the confusion matrix graphs (Figures 5 and 7), it is observed that that N is more noticeable compared to the remaining beats, also V and S beats are remarkable than F. It exposes that their ratio is misbalancing, but the proposed models classify each category properly without any biasing.

The article "An Effective and Lightweight Deep Electrocardiography Arrhythmia Recognition Model Using Novel Special and Native Structural Regularization Techniques on Cardiac Signal" was retracted in 2023. Reasons: unreliable results or conclusions; concerns about the data; concerns about the peer review; concerns about the citations.

This expresses the generalization of the developed models and a solution of data imbalance problem. From the comparison (Table 6), it is also observed that all 2D CNN approaches deliver better results compared to 1D CNN. So, the transformation of sequential beat information into their corresponding beat images is a promising strategy. The R-R intervals or R-peaks, duration, and amplitude of the QRS are highly sensitive to the dynamic and morphology features of complex ECG. The transformation-based method reduces the problem of strict time alignment; it ignores the scoring of fiducial points of heartbeats. The nonlinear and nonstationary characteristics of ECG heartbeats due to the episodic electrical conduction of heart are the major factors behind the facing of such sensitivity. The developed models extract the desirable activation on intensity, edge, and shape of peak of our preprocessed beat images. Background is not a big deal in this study because extracted beat is appeared only at a small portion of the whole image. The peaks are more crucial factor due to the describing of both P-wave shape and R-R intervals at a time. The satisfactory performance of developed models represents the learned features from the images are well correlated and embedded with the desired classes in respect to the high dimensional (mapped in two dimension) feature space, which is more obvious from the confusion matrix graphs and evaluated matrices. Now we will discuss the issues why our proposed models provide the satisfactory findings in arrhythmia recognition. First, CNNs models learn the dominant features from its first convolution layer and finally it is investigated with the resulted classifier. Second, the most crucial stage of the experiments is segmenting and transforming ECG signals into the corresponding beat images, the work is performed with a developed python module following a well-known and effective R-peak detection algorithm [65]. Third, AlexNet and VGGNet architecture have some inspirable benefits compared to other CNN architectures such as easy GoogleNet, ResNet, DenseNet, and especially less parameters are required to train the models and result is lightweight of model. Fourth, because of using some diverse mechanisms such as early stopping [59] that helps to stop over-fitting of the models, weighted random sampler [58] for reducing the class imbalance problem of the samples, Adam optimizer [38] for handling the minimum validation loss and quick training, on-the-fly augmentation [61], stratified evaluation strategy for ensuring the samples from each class to each fold, and reducing the effect of the class imbalance problem [62, 63].

The article "An Effective and Lightweight Deep Electrocardiography Arrhythmia Recognition Model Using Novel Special and Native Structural Regularization Techniques on Cardiac Signal" was retracted in 2023. Reasons: unreliable results or conclusions; concerns about the data; concerns about the peer review; concerns about the citations.

In this study, we experimented and analyzed the performance of our proposed models only on the ECG arrhythmia data as the input of models for arrhythmia recognition. But the models could be employed for other categories of data such as HomePap, sleep-EDF, and sleep heart health study (SHHS) as the input of proposed models for analyzing the sleep disorders. For example, a deep learning approach with 2D CNN is addressed by Erdenebayar et al. for automatic detection of sleep apnea (SA) events from ECG signal recordings by an Embla N70 0 0 amplifier device (Embla System Inc., U.S.A.) at the Samsung Medical Center (Seoul, Korea) and demonstrated good results [80]. Recently, deep learning has also proved its potentiality applications in all physiological signals such as electroencephalogram (EEG), electromyogram (EMG), and 2D medical imaging [81]. Different neurological diseases such as epilepsy, Parkinson's disease (PD) [82], and Alzheimer's disease (AD) could be easily diagnosed with the EEG signals from a patient taking the benefits of 2D CNN models. For example, a novel 2D CNN model is presented by Madhavan et al. [83] for identifying the focal epilepsy from Bern-Barcelona EEG database and received the satisfactory results, where time-series EEG signals are transformed into 2D images with Fourier synchro squeezing transform (FSST) and wavelet SST (WSST) and evaluated on both cases. In addition, with EEG signals, these diseases could also be detected from the speech data [26, 84]. EMG signals are widely used in human activity and hand gesture recognition, nowadays which are more interesting for rehabilitation robots, artificial intelligence robots, active prosthetic hands, and entertainment robots as well. Besides, it is also used to diagnosis several neuromuscular diseases such as ALS (amyotrophic lateral sclerosis) because of containing some brain information [85]. Zhai et al. [86] proposed a 2D CNN model to recognize the patterns from surface electromyography (sEMG) signals of NinaPro publicly available database for controlling the upper limb neuro prosthetic and achieved better findings compared to a traditional method. Beyond the disease identification, with the preprocessing of raw information, 2D CNN could also be employed in others field such as detecting the faulty sensors in array antennas [87, 88]. Therefore, our developed models are a good prospect for the researchers who work in deep learning for identifying signal patterns.

The article "An Effective and Lightweight Deep Electrocardiography Arrhythmia Recognition Model Using Novel Special and Native Structural Regularization Techniques on Cardiac Signal" was retracted in 2023. Reasons: unreliable results or conclusions; concerns about the data; concerns about the peer review; concerns about the citations.

The lightweight of our proposed models compared to the state-of-the-art methods expresses the strength of models to deploy in real-life applications, as shown in Table 7. Small model size indicates better model efficiency. In this study, the efficiency of the proposed Deep-NSR model is too attractive compared to Deep-SR, because the total learnable parameter is drastically reduced in Deep-NSR. So, the Deep-NSR could be easily deployed in practical application to diagnose arrhythmia from the ECG signal. This result is mainly due to its design strategy. Saadatnejad et al. [89] proposed and experimented a novel lightweight deep learning approach on the wearable devices with a confined capacity for the continuous monitoring of cardiac rhythm. The measurements on various hardware platforms demonstrate that their proposed algorithm fulfills the requirements for continuous monitoring of heart rhythm in real time. This is an inspiration for us to deploy our proposed models especially Deep-NSR in real-life applications in future.

When it comes to the limitations of our proposed work, we must first take into account that our arrhythmia recognition method is only tested on publicly available datasets, no real-time data/clinical data are used for testing, but the data in MIT-BIH arrhythmia database are collected under various environmental circumstances, and devices in real time with different degrees consider various interference issues. The dataset uses standard data storage format and all data are labeled by the professional physicians. So, the dataset is more reliable data source for testing the model. Second, we have followed intra-patient paradigm in this study, where the same patient heartbeats are likely to arrive both in training and testing sets. This circumstance may lead the biased results. The patient-specific study could be the solution of the challenge. Third, our used dataset is publicly available, which is small in scale. Deep learning models consist of numerous numbers of layers with huge learnable parameters. They process the data repeatedly to acquire the optimal number of parameters during training; as a result, it may face the over-fitting problem with the small volume of datasets. This challenge could be addressed to employ the transfer learning technique [90] in the model that is trained on large volume of data previously. In addition, comprehending a relationship between the feature extraction and fundamental physiology is very important to recognize the specific disease. So, feature-based diagnosing is an interesting field to study in future.

The article "An Effective and Lightweight Deep Electrocardiography Arrhythmia Recognition Model Using Novel Special and Native Structural Regularization Techniques on Cardiac Signal" was retracted in 2023. Reasons: unreliable results or conclusions; concerns about the data; concerns about the peer review; concerns about the citations.

### 3.3. Open Challenges and Opportunities of Deep Learning Methods in ECG Data

In spite of great successes of deep learning in recognition and detection such as learning the important features, it faces several challenges: first, high computational complexity is required for model training due to the deficiency of powerful hardware [91], so it is more feasible to utilize the deep learning methods in offline processing to diagnose the cardiac arrhythmias. Using the high-level API (application programming interface) data frame provided by structured streaming platform, where fast SQL (Structured Query Language) functions on streaming data are implemented, could be a solution of overcoming this challenge of deep learning methods for online diagnosis with less delay. Generally, the computational complexity of a deep learning method depends on the required floating-point operations for processing that model, where there is a strong correlation among the floating-point operations, energy consumption (*R*^2^ = 0.9641, *p*– value < 0.0001), and inference time (*R*^2^ = 0.8888, *p*–value < 0.0015) of a CNN model. The real inference time of a deep learning method depends on the different parameters including compiler optimization, hardware platform, and used APIs to implement the model [92]. Besides, PyTorch provides optimized performance, memory usage, and energy consumption using CUDA and CUDNN with our used graphics processing unit (GPU, NVIDIA) [75]. In our experiments, the complete total computational time of Deep-SR was 451 minutes 1 second using the hardware configuration indicated in Section 2.5, while the testing computation time for a single image was 0.2769 second. On the other hand, the total computational time of Deep-NSR was 379 minutes 7 seconds, while the testing computation time for a single image was 0.2328 second. The computation time will be varied with the changing of hardware configuration of used PC. We see that the testing computation time in Deep-NSR model is less than Deep-SR, which indicates that Deep-NSR model will be more suitable to deploy in resource-constraint devices such as mobile phone, portable/wearable healthcare devices compared to Deep-SR. The occupied memory space for Deep-SR was 16.92 MB, while it was 11.49 MB for Deep-NSR, which also expresses that Deep-NSR model will be more effective to deploy in resource-constraint devices compared to Deep-SR. However, both models outperform the state-of-the-art models in the sense of performance and model size, depicted in Tables 6 and 7. So, both could be chosen to deploy in real-life applications such as resource-constraint devices and offline diagnosis in medical and clinics. Indeed, deep learning methods demand more computing resource compared to machine learning-based techniques for real-time processing, and hence these are slower [93]. Second, interpretability; it is hard to understand the reasons for human beings why a particular result is received by a deep model compared to traditional machine learning algorithms, because the deep learning models are usually considered as the black box models with huge learnable parameters. This challenge has become more severe in clinical tasks because diagnosis is not perceptible by physicians without any interpretation. To tackle the challenge, two directions are worth noted, (i) replacing a complex model by relatively a simple model, and (ii) one can add attention mechanism on the hidden layers or imitate neuron connection concepts from the tree-based model. Third, efficiency; it is difficult to deploy the big deep models into the portable healthcare devices for real-life applications. In this case, promising direction is lightweight deep model, or model compression technique such as knowledge distillation, weight sharing, and quantization. Fourth, integration with expert features; it is difficult to integrate a trained deep model with the existing expert knowledge/features. To tackle the issue, (i) one can use domain expert knowledge for designing the deep models, and (ii) coining or explicitly extract the latent embedding features from the deep models. Then one easily assembles deep and expert features and makes the traditional machine learning methods from them. Fifth, noise robustness; deep learning methods automatically extract all features from ECG signals including the various categories of real-world noises such as motion artifacts, baseline wander, electrode contact, and power line interference appeared in it, which leads to incorrect results. The issue could be something resolved by using a de-noising/filtering technique before fitting data into the input of deep models, but some valuable information may be omitted in this way [94]. So, we have not performed any de-noising/filtering technique on the raw data in our study. In our experiments, we have used MIT-BIH arrhythmia database, where ECG raw data contain several real-world noises and filtered with band-pass filter at 0.1100 Hz [64]. Recently, de-noising autoencoder (DAE), sparse autoencoder (SAE), contractive autoencoder (CAE), and generative adversarial network (GAN) are some widely used promising techniques to remove such suspected noises appeared in ECG signals. In addition to above, one more challenge of deep learning methods is the lack of availability of training data, because large volume of data are required during training the models to handle the over-fitting problem. Transfer learning techniques could recover this challenge at some extends. Finally, we should tell that the major failure case of our proposed models along with the facing challenges mentioned above is the inability to classify other categories of images properly available in real worlds beyond the ECG beat images as well as identify of all beat images correctly, which is depicted in Figures 5 and 7 (confusion matrixes for both models). However, deep learning, especially CNN-based methods are promising for diagnosing various cardiovascular diseases in offline and online.

The article "An Effective and Lightweight Deep Electrocardiography Arrhythmia Recognition Model Using Novel Special and Native Structural Regularization Techniques on Cardiac Signal" was retracted in 2023. Reasons: unreliable results or conclusions; concerns about the data; concerns about the peer review; concerns about the citations.

## 4. Conclusion and Future Works

The automatic arrhythmia recognition with machine learning algorithms has gained its importance day by day since it helps the experts to diagnose cardiovascular diseases easily, which are seen in ECG signals. In this work, the received classification performances for four cardiac rhythms on both models surpassed the state-of-the-art models that represent the better effectiveness of the proposed models. Importantly, the UAF_1_ for both models indicated that the proposed models were more generalized for imbalance classes. The lightweight of Deep-NSR model narrates its better efficiency compared to the state-of-the-art models. As such, it could be easily deployed in real-life applications in deep learning approaches. Moreover, the proposed models would be more applicable with the different amplitudes and sampling rates in various ECG devices. The present study employed ECG signals from a single lead. Signals from multiple leads will be studied in future to more enrich the experimental cases. Furthermore, we have also planned to work on such interesting, related directions as (i) adapting the models for other diseases like sleep apnea with the corresponding datasets related to ECG signals, (ii) expanding the adaptation scope of our proposed models for EEG and EMG signal-related dataset, and (iii) verifying the performance of proposed models with own developed sensor/real-time data.

## Figures and Tables

**Figure 1:** Workflow diagram of our proposed method for ECG arrhythmia classification.

**Figure 2:** An end-to-end internal layer architecture of the proposed Deep-SR model.

**Figure 3:** The layered end-to-end internal architecture of the proposed Deep-NSR model.

**Figure 4:** Normal and seven ECG arrhythmia beats. N, normal beat; V, premature ventricular contraction (PVC) beat; A, atrial premature contraction (APC) beat; R, right bundle branch block (RBB) beat; L, left bundle branch block (LBB) beat; P, paced beat; E, ventricular escape beat (VEB); and !-ventricular flutter wave (VFW) beat.

The article "An Effective and Lightweight Deep Electrocardiography Arrhythmia Recognition Model Using Novel Special and Native Structural Regularization Techniques on Cardiac Signal" was retracted in 2023. Reasons: unreliable results or conclusions; concerns about the data; concerns about the peer review; concerns about the citations.

**Figure 5:** Confusion matrix for the proposed Deep-SR model.

**Figure 6:** Stratified five-fold cross-validation results for arrhythmia recognition for the proposed Deep-SR model: (a) Average accuracy, UAR, and UAF_1_; (b) Training and testing loss curve.

**Figure 7:** Confusion matrix for the proposed Deep-NSR model.

**Figure 8:** Stratified five-fold cross-validation results for arrhythmia recognition for the proposed Deep-NSR model: (a) average accuracy, UAR, and UAF1; (b) training and testing loss curve.

**Table 1:** The internal architecture of the proposed Deep-SR model with its relevant hyperparameters. Here, ReLU is used after each convolution layer and BN is used after each ReLU and dropout; fully connected and softmax layers are not shown.

Layer name	Output size	Kernel size	# Filters	Stride
Conv2d-1	62 × 62	5 × 5	32	2
MaxPool2d-4	30 × 30	3 × 3	1	2
Conv2d-5	28 × 28	3 × 3	64	1
Conv2d-8	26 × 26	3 × 3	128	1
Conv2d-11	24 × 24	3 × 3	256	1
AvgPool2d-14	11 × 11	3 × 3	1	2
Conv2d-15	9 × 9	3 × 3	512	1
AdaptiveAvgPool2d-18	1 × 1	9 × 9	1	—

**Table 2:** The internal architecture of the proposed Deep-NSR model with its relevant hyperparameters. Here, ReLU is used after each convolution layer and BN is used after each ReLU and dropout; fully connected and softmax layers are not shown.

Layer name	Output size	Kernel size	# Filters	Stride
Conv2d-1	62 × 62	5 × 5	32	2
MaxPool2d-4	30 × 30	3 × 3	1	2
Conv2d-5	28 × 28	3 × 3	64	1
Conv2d-8	26 × 26	3 × 3	128	1
Conv2d-11	24 × 24	3 × 3	256	1
AvgPool2d-14	11 × 11	3 × 3	1	2
Conv2d-15	9 × 9	3 × 3	8	1
AdaptiveAvgPool2d-18	1 × 1	9 × 9	1	—

**Table 3:** A summary of all metrics from the confusion matrix of Deep-SR model.

Accuracy (%)		Precision (%)		Recall (%)		F_1score_ (%)	
N	99.94	N	99.99	N	99.94	N	99.97
S	99.98	S	99.78	S	99.67	S	99.63
V	99.94	V	99.27	V	99.94	V	99.62
F	99.99	F	99.20	F	99.84	F	99.52
Average	99.96	Average	99.56	Average	99.85	Average	99.67

**Table 4:** The comparison of evaluation matrices, validation loss, and size of both models.

Evaluation matrices/validation loss/learnable parameters/model size	Proposed Deep-SR model	Proposed Deep-NSR model
Overall testing accuracy	0.9993	0.9996
Unweighted overall recall	0.9985	0.9998
Unweighted overall F_1_score_	0.9971	0.9987
Minimum validation loss	0.0117	0.0200
Learnable parameters	1573156	**399656**
Model size	16.92 MB	**11.49 MB**

**Table 5:** A summary of all metrics from the confusion matrix of Deep-NSR model.

Accuracy (%)		Precision (%)		Recall (%)		F_1score_ (%)	
N	99.96	N	100	N	99.95	N	99.98
S	99.99	S	99.89	S	100	S	99.94
V	99.96	V	99.47	V	99.94	V	99.72
F	99.99	F	99.68	F	100	F	99.84
Average	99.98	Average	99.76	Average	99.97	Average	99.87

**Table 6:** Comparison with the state-of-the-art models.

Classifier type	Works	#Class category	Accuracy (%)	Recall (%)	F_1score_
2D CNN (Prop.)	Deep-SR	4	**99.93** ^*∗∗*^ **99.96** ^*∗∗*^ 98.92^*∗*^ 99.11^*∗∗*^	**99.85** ^*∗∗*^ **99.98** ^*∗∗*^ 97.26^*∗*^ 97.91^*∗∗*^	**99.71** ^*∗∗*^ **99.87** ^*∗∗*^ 98.00^*∗*^ 98.00^*∗∗*^
2D CNN (Prop.)	Deep-NSR	4			
2D CNN	Ullah et al. [52]	8			
2D CNN	Jun et al. [53]	8	99.05^*∗*^ 98.90^*∗∗*^	97.85^*∗*^ 97.20^*∗∗*^	—
2D CNN	Alex Net [53]	8	98.85^*∗*^ 98.81^*∗∗*^	97.08^*∗*^ 96.81^*∗∗*^	—
2D CNN	VGG Net [53]	8	98.63^*∗*^ 98.77^*∗∗*^	96.93^*∗*^ 97.26^*∗∗*^	—
2D CNN	Izci et al. [54]	5	99.05^*∗*^	—	—
2D CNN	Huang et al. [51]	5	99.00^*∗*^	—	—
2D CNN	Lu et al. [50]	5	96.00^*∗*^	96.80^*∗*^	96.40^*∗*^
1D CNN	Zubai et al. [47]	5	92.70^*∗*^	—	—
1D CNN	Ullah et al. [52]	8	97.80^*∗*^	—	—
1D CNN	Huang et al. [51]	5	90.93^*∗*^	—	—
1D CNN	Li et al. [48]	5	97.50^*∗*^	—	—
1D CNN	Lu et al. [50]	5	94.00^*∗*^	96.00^*∗*^	95.19^*∗*^
TQWT + SVM	Jha et al. [12]	8	99.27^*∗*^	—	—
CEEMDAN + PCA + ANN	Abdalla et al. [13]	5	99.90^*∗*^	—	—
LBP, HOS + Ensemble SVM	Mondéjar-Guerra et al. [14]	4	94.50^*∗*^	—	—

^*∗∗*^With augmentation on-the-fly or manual, ^*∗*^without augmentation, TQWT-tunable Q-wavelet transform, and CEEMDAN-complete ensemble empirical mode decomposition with adaptive noise.

The article "An Effective and Lightweight Deep Electrocardiography Arrhythmia Recognition Model Using Novel Special and Native Structural Regularization Techniques on Cardiac Signal" was retracted in 2023. Reasons: unreliable results or conclusions; concerns about the data; concerns about the peer review; concerns about the citations.

**Table 7:** Comparison with the existing models.

Classifier type	Works	#Class category	Model Size(MB)	#Learnable Parameters
2D CNN (Proposed)	Deep-SR Model	4	**16.92**	1573156
2D CNN (Proposed)	Deep-NSR Model	4	**11.49**	399656
2D CNN	Ullah et al. [52]	8	49.91	1557016
2D CNN	Jun et al. [53]	8	81.67	1149272
2D CNN	Alex Net [53]	8	34.05	947092
2D CNN	VGG Net [53]	8	84.66	7639440

## Data Availability

The data used to support the findings of the study are available from the corresponding authors upon request.
